# The Effect of High-Speed Power Training on Physical Frailty in Older Adults: Effect of a Visual-Guided Exercise Program in South Korean Rural Areas

**DOI:** 10.1155/2023/8912846

**Published:** 2023-06-02

**Authors:** Dong Hyun Yoon, Jin-Soo Kim, Su Seung Hwang, Dong Won Lee, Wook Song

**Affiliations:** ^1^Department of Rehabilitation Medicine, Seoul Metropolitan Government Boramae Medical Center, Seoul, Republic of Korea; ^2^Institute on Aging, Seoul National University, Seoul 08826, Republic of Korea; ^3^Exercise Medicine Research Institute, Edith Cowan University, Joondalup, WA 6027, Australia; ^4^School of Medicine and Sciences, Edith Cowan University, Joondalup, WA 6027, Australia; ^5^Health and Exercise Science Laboratory, Department of Physical Education, Institute of Sports Science, Seoul National University, Seoul 08826, Republic of Korea

## Abstract

**Objective:**

Exercise has been shown to be an effective intervention; the difficulty still lies in providing exercise programs to the older adults in rural areas. Therefore, this study aimed to examine the effects of a 12-week exercise program provided with visual guidelines (prerecorded video) on frailty among older adults in rural areas.

**Methods:**

Fifty participants (71.7 ± 4.9 years) from 5 different rural areas were recruited and divided into two groups: the exercise group (EX, *n* = 24 (male: 8, female: 18)) and the control group (CON, *n* = 26 (male: 7, female: 17)). With the commencement of the exercise intervention, a prerecorded high-speed power training program for frail older adults was distributed to the EX group. A new prerecorded exercise program was delivered to the EX group every 4 weeks. Frailty status was diagnosed with Fried's criteria before and after the intervention. Muscle strength was measured in the upper and lower limb strength (hand-grip strength and leg extension and flexion), and physical function was measured using a short physical performance battery and gait speed. Fasting blood was collected before and after the intervention and analyzed for blood lipid profile.

**Results:**

After 12 weeks of the intervention period, a significant difference in frailty status (*P* < 0.01) and score (*P* < 0.01) favoring the EX group was observed. Physical functions (gait speed (*P*=0.01) and time for sit to stand (*P* < 0.01)) were significantly improved in the EX group with a significant increase in knee extensor strength (*P* < 0.01). A significant difference in serum high-density lipoprotein levels favoring the EX group (*P*=0.03) was also observed.

**Conclusions:**

This study confirmed the positive effect of a visual-guided exercise program on older adults' residents in rural areas and provided alternative methods to effectively provide exercise program for the older adults with limited resources.

## 1. Introduction

Frailty refers to physiological and physical impairment resulting from aging-related deterioration of overall function [1]. This includes impaired neuroendocrine function and immunity, as well as reduced muscle mass, muscle strength, and physical activity, leading to a reduced appropriate response to external stress and increasing the risk of disease morbidity and disability [1, 2]. As a result, the incidence of adverse health outcomes in frailty is twice that in prefrail status [3], resulting in hypofunction, insensibility, loss of appetite, and ultimately death, regardless of the presence of illness [1]. Therefore, early diagnosis and intervention (treatment) that could delay aspects of frailty are crucial in improving health in the older adults [2, 4].

Age-related impairment in skeletal muscle causes an imbalance of muscle protein synthesis and breakdown, leading to a substantial loss of skeletal muscle mass [5]. Furthermore, a pronounced muscle power loss is shown with aging and is strongly associated with reduced physical function in older adults [1, 6]. As such, while multiple intervention methods are available, exercise has shown its effectiveness in alleviating frailty [1], owing to its capacity to improve the production and use of energy in the entire body system and enhance physical function [4, 7, 8]. In a clinical trial, Fiatarone et al. demonstrated improvement in physical function (gait speed and skeletal muscle power) and skeletal muscle cross-sectional area with a 10-week supervised resistance exercise in older adults with frailty [7]. Furthermore, a large, randomized trial LIFE study in 2014 reported reduced mobility disability over 2.6 years of combined (resistance and aerobic) exercise among older adults with a risk of disability [8].

Although the effectiveness of exercise in alleviating frailty is well documented, exercise intervention in the studies consisted of supervision, limiting its application to older adults, especially in rural areas [9]. Moreover, the lack of resources, such as exercise facilities and equipment, for exercise in rural areas further limits this population from engaging in exercise [10]. Particularly for resistance exercise, professional instructors, facilities, and equipment are critical; it is essential to determine a way to provide exercise treatment safely and effectively in rural areas using available resources. As the visual-guided exercise program based on video has demonstrated their effectiveness in improving physical function and activity in frail older adults [11, 12], it could potentially be a safe and effective method for delivering the resistance exercise program in older individuals in rural areas with its capacity to provide visual and linguistic instruction [13]. As such, we examined the effect of a prerecorded visual-guided high-speed power training program on frailty phenotypes in the older population in rural areas. Furthermore, as frailty is associated with risk factors for cardiovascular disease [14], we also examined the blood lipid profile and skeletal muscle mass to further examine the potential contribution of exercise in reducing risk factors for cardiovascular disease in this population.

## 2. Methods

### 2.1. Participants and Group Assignment

Hundred and fifteen older adults from 5 different rural villages in the Republic of Korea were screened for participation, and their progression through the study is shown in Figure 1. Inclusion criteria included the following: age ≥ 65 years, ambulatory with or without an assistive device, and able to perform frailty criteria testing. Older adults who were hospitalized and had a Mini-Mental State Examination (MMSE) score of 18 or less were excluded. Due to the absence of a community center and the agriculture pattern of different rural villages, random assignment of the group was not possible; as a result, 37 older adults from 3 rural villages were assigned to the exercise group (EX), and 40 older adults from 2 rural villages were assigned to the control group (CON). During the intervention, a total of 27 participants withdrew (EX, *n* = 13; CON, *n* = 14), resulting in 24 participants from the EX group and 26 participants completing the trial (Figure 1). Ethical approval was obtained from the Institutional Review Board before the commencement of the trial, and written consent was obtained from each participant.

### 2.2. Video-Based Visual-Guided Exercise Program

For exercise intervention, the participants were provided with a video-recorded exercise program and asked to follow exercise twice a week for 12 weeks. The 45-minute video-recorded exercise consisted of a 5-minute warm-up, 35 minutes of elastic-band-based high-speed power training, and a 5-minute cool down. An elastic band (Hygienic Corporation, USA) with an appropriate intensity for each individual was provided based on their baseline strength testing. The exercise consisted of 5–7 different resistance exercises (3 sets, 12 repetitions) involving large muscle groups focusing on the speed of concentric motion with a slow eccentric motion. The video provided the exact timing of the concentric phase (as fast as possible and pause for approximately 1 second) and eccentric phase (2 seconds) [15, 16] with visual and linguistic instruction. The prerecorded exercise program was distributed at the local community center, and supervised familiarisation sessions were provided during the first two weeks of intervention. A new video was distributed every four weeks to increase the volume and intensity of exercise. With the distribution of the new exercise video, the rating of perceived exertion (RPE; 6–20 Borg scale) was assessed to evaluate the exercise session.

### 2.3. Frailty Assessment

Physical frailty was assessed according to the criteria introduced by Fried et al. in 2001 [2]. These criteria grade frailty in three categories, frail (3 or more phenotypes), prefrail (1 or 2 phenotypes), and robust (no phenotype), by evaluating the following five phenotypes for physical frailty [2]:

1. Shrinking: low body mass index (BMI < 18.5 kg/m^2^), self-reported unintentional weight loss of 4.5 kg in the past year, or ≥ 5% body weight loss in the past year.
2. Weakness: grip strength in the lowest 20%, adjusted for gender and body mass index
3. Poor endurance and energy: self-report of exhaustion by two questions in the Center for Epidemiological Studies-Depression Scale (CES-D) [17]
4. Slowness: gait speed in the slowest 20%, adjusted for gender and height
5. Low activity: low physical activity determined by the International Physical Activity Questionnaire (IPAQ)

### 2.4. Body Composition and Rectus Femoris Thickness

Body composition, including body weight, total mass, lean mass, fat mass, and BMI, was measured using bioelectric analysis (Inbody370, Seoul, Korea), and height was measured using a manual extensometer before and after a 12-week intervention. The thickness of the quadriceps muscle was measured before and after 12 weeks using portable ultrasonography (BodyMetrix BX-2000, IntelaMetrix Inc., CA, USA) with a standard 2.5 MHz probe and A-mode transducer. However, due to the limitation of portable devices, only the thickness of the rectus femoris was measured and analyzed. Measurements were taken from each subject with the lower limb extended and relaxed after resting for 10 to 15 minutes to allow fluid shifts to occur. The probe position for rectus femoris measurements was the same as that used in previous studies [18, 19]. The image was analyzed using the portable ultrasonography manufacturer-providing software (BodyView, IntelaMetrix Inc., CA, USA).

### 2.5. Muscle Strength

Hand-grip strength was measured in Newton (N) using a hand-held dynamometer based on strain gauge sensors (Takei Scientific Instruments, Niigata, Japan) before and after the intervention. Furthermore, leg muscle strength was measured by using a hand-held portable dynamometer (model 01163, Lafayette Instrument Company, Lafayette, Ind., USA). The participants were asked to perform two maximal contractions of 5–10 seconds for each muscle group [20] in a sitting position, and a 60-second rest was provided between each contraction.

### 2.6. Physical Function

A short physical performance battery (SPPB) was used to assess balance, walking, strength, and endurance. Each test receives a performance score, with a total of 12 points comprising the chair stand test (4 points), balance test (4 points), and gait speed test (4 points) [21].

### 2.7. Blood Assessment and Analysis

Blood assessments and analysis were undertaken by the commercial biological sample collection and analysis service (GC Cell, Yongin-si, Korea). On the morning of the test day, 20 ml of blood was collected after 12 hours of fasting in a serum separating tube (SST) and transferred to the certified laboratory (GC Cell, Yongin-si, Korea) in an icebox (4°C). Serum levels of total glucose, total cholesterol, triglyceride (TG), low-density lipoprotein (LDL), and high-density lipoprotein (HDL) were measured on the same day.

### 2.8. Statistical Analyses

The statistical analyses were performed using SPSS (version 23.0, IBM Corporation, Chicago, IL, USA). The normality of the data was tested using the Shapiro–Wilk test and the Q-Q plot. Analyses included standard descriptive statistics and two-way (group *x* time) repeated measures analysis of variance (ANOVA). Follow-up tests were performed if the interaction or main effect for time was significant (paired *T*-test). Tests were two-tailed, with an alpha level of 0.05 as the statistical significance criterion.

## 3. Results

### 3.1. Participant Characteristics

Participant characteristics are summarized in Table 1. There was no significant difference in age, frailty criteria, anthropometrics, and body composition. Notably, there was no difference in the percentage of individuals with three different categories of frailty in the EX and CON groups.

### 3.2. Frailty

Three categories of frailty, robust, prefrail, and frail, were converted to 1 (robust), 2 (prefrail), and 3 (frail) and analyzed. As a result, a significant difference was observed in the group by time analysis of mean frailty status (*P* < 0.01) (Table 2). Postanalysis showed a significant reduction after a 12-week exercise intervention in the EX group (*P* < 0.01) but unchanged in the CON group. Importantly, the number of participants categorized as frail reduced from 5 to 0 in the EX group. On the contrary, the number of frail participants in the CON group increased from 3 to 8. Mean frailty scores based on Fried et al. [2] were also significantly reduced in the EX group after the 12-week exercise intervention (pre: 1.45 ± 1.28 vs. post: 0.87 ± 0.79; *P* < 0.01) but increased in the CON group (pre: 1.46 ± 1.20 vs. post: 2.19 ± 0.63; *P* < 0.01).

### 3.3. Body Composition and Blood Lipid Profile

No significant changes in body composition (weight, skeletal muscle mass, fat mass, and BMI) were observed (Table 3). In addition, no changes were observed in the thickness of the rectus femoris (Table 3). Blood lipid profile was also examined, and no changes were observed in serum glucose, triglyceride, total cholesterol, and LDL. Still, a significant difference was observed in HDL favoring the EX group. Postanalysis revealed that the difference observed in HDL was due to a significant reduction in HDL in the CON group after the intervention period (pre: 56.35 mg/dL ± 14.62 vs. post: 53.08 mg/dL ± 12.60; *P* < 0.001) (Table 3).

### 3.4. Muscle Strength and Physical Function

For muscle strength, grip strength, knee extensor, and knee flexor were measured, and there was a significant difference in knee extensor strength favoring the EX group (*P* < 0.01) (Table 3). However, grip strength and knee flexor strength were not changed. Postanalysis demonstrated a significant increase in knee extensor strength in the EX group after 3 months of exercise intervention (pre: 70.43 Nm ± 26.18 vs. post: 84.75 Nm ± 23.64; *P* < 0.001) (Table 3). In addition, although there were no changes in SPPB score, gait speed (*P*=0.04) and time for sit to stand (*P*=0.05) showed a significant difference, favoring the EX group. Postanalysis also demonstrated a significant reduction in gait speed (pre: 5.54 sec ± 2.24 vs. post: 5.30 sec ± 1.81; *P* < 0.01) and time for sit to stand (pre: 10.78 sec ± 3.47 vs. post: 8.01 ± 1.86; *P* < 0.01) in the EX group after the 3-month exercise intervention.

## 4. Discussion

To our knowledge, this is the first two-armed study to evaluate the effect of the visual-guided exercise program on frailty levels in older adults in the rural areas of the Republic of Korea. We examined the frailty score based on criteria presented in the report by Fried et al. [2] and showed a significant reduction in frailty status and scores in the EX group compared with the CON group. In addition, although the body composition did not change, a significant difference in blood profile (serum HDL levels) and lower body strength favoring the EX group was observed after 12 weeks. Lastly, gait speed and time for sit to stand were significantly reduced in the EX group; however, the SPPB score did not improve after exercise intervention.

Frailty is an important factor determining the quality of life and life span of older individuals. As such, it has been reported that early diagnosis and intervention in the clinical approach are critical for healthy aging in the older adults [22]. The detailed categorization of frailty was performed by Fried et al. in 2001 [2], and since then, multiple studies have demonstrated the efficacy of exercise in improving frailty status [7, 8, 23]. Although these studies observed the improvement of physical function by conducting in-clinic supervised exercise [7, 8, 23], whether exercise could reverse physical frailty in older adults in rural areas could not be evaluated due to limited accessibility. Moreover, although a higher prevalence of frailty has been reported previously, exercise intervention is not well implemented in rural areas due to limited exercise facilities, equipment, and expert exercise physiologists [10]. As such, as important as evaluating the effect of exercise on frailty in the older adults in rural areas, determining an effective method to deliver the exercise program is critical to benefit older adults in rural areas.

In line with this, we delivered an exercise program for 12 weeks with a video by providing a new video every 4 weeks to adjust the intensity and volume of exercise and demonstrated a significant reduction in frailty scores and status in older adults living in rural areas. This result was similar to that of previous studies by Kim et al. [24], Fairhall et al. [3], and Yu et al. [23], which used supervised exercise intervention to examine the effect of exercise in older adults and reported a reduction of frailty and improved physical function. Furthermore, the improvement of physical function, such as gait speed and time for sit to stand, was demonstrated in the present study as was reported in previous studies which examined the effect of video exercise program on physical function in older women and older adults with the locomotive syndrome [11, 12]. Although the effectiveness of two different exercise delivery methods (direct supervision vs. video exercise program) could not be compared, the outcome from the present study is important for those with limited access to direct supervision by demonstrating the effect of visual-guided exercise program in reducing frailty.

The present study also examined the changes in body composition, including muscle thickness, and muscle strength, after 12 weeks. However, we did not observe differences in body composition, including body weight and skeletal muscle mass. This was inconsistent compared to previous reports that investigated the effect of exercise on body composition in older adults [25, 26], and this inconsistency was further shown by demonstrating no changes observed in skeletal muscle thickness (rectus femoris). This might be caused by a difference in exercise modality implemented in the studies. Although the mechanistic explanations for discreet body composition (especially muscle hypertrophy) resulting from different exercise modalities are currently unknown, the exercise we implemented (high-speed power training) is known to increase muscular power having a greater impact on physical function compared to traditional resistance exercise [15, 27]. This might have played a role in different outcomes in body composition compared to the previous studies. In contrast, we observed a consistent increase in skeletal muscle strength (knee extensor) compared to previous studies [15, 27] after 12 weeks, confirming the efficacy of video-delivered high-speed power training in increasing muscle strength in older adults in rural areas, along with a substantial increase in physical functions that are highly related to lower body strength.

In addition, the blood lipid profile was also measured before and after the 12-week intervention to examine the potential contribution of exercise to the risk of cardiovascular disease. It has been shown that older adults with frailty have worsened cardiovascular risk profiles, such as low HDL, hypertension, and high waist circumference, compared with those who are not frail [14]. In addition, recently, the triglyceride (TG)-HDL ratio has been shown to be associated with cardiovascular disease risk [28]. Although a significant alteration of TG-HDL ratio in our cohort after the exercise program was not observed, we showed a significant change in serum HDL levels over 12 weeks of intervention favoring the EX group (significant reduction in the CON group and increased trend in the EX group), suggesting that exercise has a potential impact on the risk of cardiovascular diseases by sustaining serum HDL levels in our cohort and further contributing to healthy aging.

The present study has strength worthy of noting. This study examined the effect of exercise on frailty in older adults in rural areas without adequate resources for executing exercise programs (equipment and human resources). This study may provide valuable initial data for developing interactive remote exercise programs for older adults with limited resources. Moreover, as the current social paradigm avoids direct personal contact owing to COVID-19, the present study showed an alternative method to deliver exercise to the older adults to improve frailty. Moreover, this study also has limitations that need to be addressed to reduce the bias of our outcomes. The EX and CON groups were not randomly assigned due to the different agricultural patterns of different villages. For example, the agriculture patterns for 3 rural villages assigned to the EX group cultivate crops requiring a short period, and 2 rural villages assigned to the CON group mainly grow fruits requiring 6 to 9 months, prohibiting us from random assignment. In addition, as all the measurements were taken in the rural villages, we could only use portable devices, prohibiting us from assessing physical measures with gold-standard methods, such as dual-energy X-ray absorptiometry and Cybex isokinetic muscle strength testing.

## 5. Conclusions

The present study provides evidence for reduced frailty status and scores with substantial improvement of physical function, specifically in gait speed and lower limb strength following a 12-week visual-guided exercise program, and provides an alternative method to deliver exercise programs to rural areas with limited resources. Furthermore, this study may provide initial data in developing remote-interactive exercise platforms that potentially contribute to healthy aging in older adults in rural areas. However, the effect of visual-guided exercise programs based on other exercise modalities needs to be examined further to provide a targeted exercise program for improving specific frail phenotypes. Lastly, additional research with randomization is also required to fully elucidate the effect of visual-guided exercise programs in improving physical functions.

## Figures and Tables

**Figure 1:** Consort diagram.

**Table 1:** Participants' characteristics at study inclusion.

	CON group (*n* = 26)	EX group (*n* = 24)	*P* value
Gender (*n*)			0.16
Male	8	7	
Female	18	17	
Age, year (mean ± SD)	71.65 ± 5.32	71.79 ± 4.42	0.41
Living alone (*n*)			
Spouse	12	12	
Alone	3	9	
Children	1	1	
Education, year (mean ± SD)	4.23 ± 4.56	5.79 ± 3.93	0.47
Conditions (*n*)			
Smoking			0.05
No	25	24	
Yes	1	0	
Alcohol			0.02
No	15	18	
Yes	11	6	
Chronic disease			0.57
No	14	15	
1>	10	9	
Job (*n*)			0.17
No	9	11	
Yes	17	13	
Frailty status (mean ± SD)	1.92 ± 0.56	2.00 ± 0.65	0.55
Robust (*n*)	5	5	
Prefrail (*n*)	18	14	
Frail (*n*)	3	5	
Frailty score (mean ± SD)	1.46 ± 1.20	1.45 ± 1.28	0.58
Body composition (mean ± SD)			
Height (cm)	152.19 ± 7.26	152.39 ± 9.22	0.96
Weight (kg)	55.10 ± 8.08	57.42 ± 7.63	0.36
Skeletal muscle mass (kg)	19.61 ± 4.11	20.08 ± 5.98	0.16
Fat mass (kg)	18.39 ± 6.20	18.07 ± 7.23	0.69
BMI (kg/m^2^)	23.83 ± 3.46	24.79 ± 3.32	0.44
Percentage of fat	33.13 ± 9.22	31.11 ± 10.98	0.75
MMSE score (mean ± SD)	23.30 ± 3.55	22.95 ± 3.38	0.76

Frailty categories (robust, prefrail, and frail) were converted to 1 (robust), 2 (prefrail), and 3 (frail), and mean and standard deviation for frailty status were calculated. BMI, body mass index.

**Table 2:** Effects of intervention on frailty score and status.

	CON group (*n* = 26)		EX group (*n* = 24)		*P* value
	Baseline	Post	Baseline	Post	
Frailty status (mean ± SD)	1.92 ± 0.56	1.92 ± 1.29	2 ± 0.65	1.58 ± 0.50^*∗∗*^	<0.01
Number of category: robust (*n*)	5	3	5	10	
Number of category: prefrail (*n*)	18	15	14	14	
Number of category: frail (*n*)	3	8	5	0	
Frailty score (mean ± SD)	1.46 ± 1.20	2.19 ± 0.63^*∗∗*^	1.45 ± 1.28	0.87 ± 0.79^*∗∗*^	<0.01
Frailty criteria					
Number of shrinking (*n*)	7	6	4	4	
Number of weakness (*n*)	16	11	14	2	
Number of exhaustion (*n*)	6	9	3	3	
Number of slowness (*n*)	2	6	5	5	
Number of low activity (*n*)	7	18	9	7	

Frailty categories (robust, prefrail, and frail) were converted to 1 (robust), 2 (prefrail), and 3 (frail) for two-way repeated measures ANOVA. ^*∗*^*P* < 0.05 compared with prefrail; ^*∗∗*^*P* < 0.01 compared with prefrail.

**Table 3:** Body composition, strength, physical function, and blood lipid profile.

	CON group (*n* = 26)		EX group (*n* = 24)		*P* value
	Baseline	Post	Baseline	Post	
Body composition and muscle thickness					
Weight (kg)	55.10 ± 8.08	55.18 ± 8.22	57.42 ± 7.63	58.38 ± 6.92	0.23
Skeletal muscle mass (kg)	19.61 ± 4.11	19.14 ± 3.84	20.08 ± 5.98	20.82 ± 4.24	0.13
Fat mass (kg)	18.39 ± 6.20	19.28 ± 5.33	18.07 ± 7.23	19.53 ± 6.41	0.72
BMI (kg/m^2^)	23.83 ± 3.46	23.29 ± 3.17	24.79 ± 3.32	24.70 ± 3.34	0.26
Percentage of fat (%)	33.13 ± 9.22	34.79 ± 7.68	31.11 ± 10.98	33.35 ± 9.45	0.82
Rectus femoris thickness (mm)	20.45 ± 5.37	22.11 ± 5.64	21.12 ± 4.59	23.80 ± 4.77	0.63
Blood lipid profile					
Glucose (mg/dL)	95.30 ± 11.00	100.00 ± 16.55	102.70 ± 35.70	101.83 ± 12.74	0.41
Triglyceride (mg/dL)	106.69 ± 45.21	137.31 ± 45.94	119.75 ± 45.21	130.75 ± 60.16	0.19
Total cholesterol (mg/dL)	181.77 ± 31.17	193.65 ± 28.20	165.88 ± 55.04	137.31 ± 45.94	0.25
Low-density lipoprotein (mg/dL)	108.42 ± 25.64	119.12 ± 27.08	98.08 ± 45.01	116.83 ± 35.97	0.35
High-density lipoprotein (mg/dL)	56.35 ± 14.62	53.08 ± 12.60^*∗∗*^	48.67 ± 18.29	53.83 ± 15.16	0.03
Triglyceride/HDL ratio	2.01 ± 0.969	2.78 ± 1.24	2.82 ± 1.53	2.83 ± 1.86	0.189
Strength					
Grip strength (kg)	23.47 ± 6.07	20.82 ± 6.27	26.70 ± 6.57	23.72 ± 5.92	0.68
Knee extensor (Nm)	64.12 ± 20.08	70.20 ± 21.48	70.43 ± 26.18	84.75 ± 23.64^*∗∗*^	<0.01
Knee flexor (Nm)	38.40 ± 11.85	44.74 ± 16.57	44.35 ± 18.74	53.73 ± 16.19	0.19
Physical function					
SPPB (score)	10.50 ± 1.42	10.53 ± 1.50	10.54 ± 1.86	10.70 ± 1.48	0.75
Gait speed (second)	4.84 ± 0.76	5.30 ± 1.02	5.54 ± 2.24	5.30 ± 1.81^*∗∗*^	0.04
Time for sit to stand (second)	11.89 ± 3.18	10.99 ± 5.17	10.78 ± 3.47	8.01 ± 1.86^*∗∗*^	0.05

The *P* values presented are the result of ANOVA analysis. Within-group analyses are presented with asterisks. ^*∗*^*P* < 0.05 compared with prefrail; ^*∗∗*^*P* < 0.01 compared with prefrail.

## Data Availability

The data used to support the findings of this study are available from the corresponding author upon request.

## Additional Points

Reduced frailty with increased physical function was shown after a 12-week visual-guided exercise program in older people in rural areas, suggesting that it can be an alternative exercise delivery method for underserved areas.

## References

[1] Angulo J., El Assar M., Alvarez-Bustos A., Rodríguez-Mañas L. (2020). Physical activity and exercise: strategies to manage frailty. *Redox Biology*.

[2] Fried L. P., Tangen C. M., Walston J. (2001). Frailty in older adults: evidence for a phenotype. *The Journals of Gerontology Series A: Biological Sciences and Medical Sciences*.

[3] Fairhall N., Sherrington C., Kurrle S. E., Lord S. R., Lockwood K., Cameron I. D. (2012). Effect of a multifactorial interdisciplinary intervention on mobility-related disability in frail older people: randomised controlled trial. *BMC Medicine*.

[4] Rodriguez-Mañas L., Fried L. P. (2015). Frailty in the clinical scenario. *The Lancet*.

[5] Wilkinson D. J., Piasecki M., Atherton P. J. (2018). The age-related loss of skeletal muscle mass and function: measurement and physiology of muscle fibre atrophy and muscle fibre loss in humans. *Ageing Research Reviews*.

[6] Casas Herrero Á., Cadore E. L., Martínez Velilla N., Izquierdo Redin M. (2015). El ejercicio físico en el anciano frágil: una actualización. *Revista Española de Geriatría y Gerontología*.

[7] Fiatarone M. A., O’Neill E. F., Ryan N. D. (1994). Exercise training and nutritional supplementation for physical frailty in very elderly people. *New England Journal of Medicine*.

[8] Pahor M., Guralnik J. M., Ambrosius W. T. (2014). Effect of structured physical activity on prevention of major mobility disability in older adults: the LIFE study randomized clinical trial. *JAMA*.

[9] Gnjidic D., Le Couteur D. G., Hilmer S. N. (2014). Sedative load and functional outcomes in community-dwelling older Australian men: the CHAMP study. *Fundamental and clinical Pharmacology*.

[10] Seo Y., Kim M., Shim H., Won C. W. (2021). Differences in the association of neighborhood environment with physical frailty between urban and rural older adults: the Korean frailty and aging cohort study (KFACS). *Journal of the American Medical Directors Association*.

[11] Vestergaard S., Kronborg C., Puggaard L. (2008). Home-based video exercise intervention for community-dwelling frail older women: a randomized controlled trial. *Aging Clinical and Experimental Research*.

[12] Hashizume H., Yoshimura N., Nagata K. (2014). Development and evaluation of a video exercise program for locomotive syndrome in the elderly. *Modern Rheumatology*.

[13] Benavent-Caballer V., Rosado-Calatayud P., Segura-Orti E., Amer-Cuenca J., Lisón J. (2016). The effectiveness of a video-supported group-based Otago exercise programme on physical performance in community-dwelling older adults: a preliminary study. *Physiotherapy*.

[14] Stewart R. (2015). Do risk factors for cardiovascular disease also increase the risk of frailty?. *Heart*.

[15] Sayers S. P., Gibson K. (2014). High-speed power training in older adults: a shift of the external resistance at which peak power is produced. *The Journal of Strength and Conditioning Research*.

[16] Yoon D. H., Lee J. Y., Song W. (2018). Effects of resistance exercise training on cognitive function and physical performance in cognitive frailty: a randomized controlled trial. *The Journal of Nutrition, Health and Aging*.

[17] Orme J. G., Reis J., Herz E. J. (1986). Factorial and discriminant validity of the center for epidemiological studies depression (CES-D) scale. *Journal of Clinical Psychology*.

[18] Lopez P., Pinto M. D., Pinto R. S. (2019). Does rest time before ultrasonography imaging affect quadriceps femoris muscle thickness, cross-sectional area and echo intensity measurements?. *Ultrasound in Medicine and Biology*.

[19] Radaelli R., Brusco C. M., Lopez P. (2018). Higher muscle power training volume is not determinant for the magnitude of neuromuscular improvements in elderly women. *Experimental Gerontology*.

[20] Muff G., Dufour S., Meyer A. (2016). Comparative assessment of knee extensor and flexor muscle strength measured using a hand-held vs. isokinetic dynamometer. *Journal of Physical Therapy Science*.

[21] Guralnik J. M., Simonsick E. M., Ferrucci L. (1994). A short physical performance battery assessing lower extremity function: association with self-reported disability and prediction of mortality and nursing home admission. *Journal of Gerontology*.

[22] Tarazona-Santabalbina F. J., Gomez-Cabrera M. C., Perez-Ros P. (2016). A multicomponent exercise intervention that reverses frailty and improves cognition, emotion, and social networking in the community-dwelling frail elderly: a randomized clinical trial. *Journal of the American Medical Directors Association*.

[23] Yu R., Tong C., Ho F. (2020). Effects of a multicomponent frailty prevention program in prefrail community-dwelling older rersons: a randomized controlled trial. *Journal of the American Medical Directors Association*.

[24] Kim H., Suzuki T., Kim M. (2015). Effects of exercise and milk fat globule membrane (MFGM) supplementation on body composition, physical function, and hematological parameters in community-dwelling frail Japanese women: a randomized double blind, placebo-controlled, follow-up trial. *PLoS One*.

[25] Bonnefoy M., Cornu C., Normand S. (2003). The effects of exercise and protein-energy supplements on body composition and muscle function in frail elderly individuals: a long-term controlled randomised study. *The British Journal of Nutrition*.

[26] Romero-Arenas S., Martinez-Pascual M., Alcaraz P. E. (2013). Impact of resistance circuit training on neuromuscular, cardiorespiratory and body composition adaptations in the elderly. *Aging and Disease*.

[27] Sayers S. P., Gibson K. (2010). A comparison of high-speed power training and traditional slow-speed resistance training in older men and women. *The Journal of Strength and Conditioning Research*.

[28] Kosmas C. E., Rodriguez Polanco S., Bousvarou M. D. (2023). The triglyceride/high-density lipoprotein cholesterol (TG/HDL-C) ratio as a risk marker for metabolic syndrome and cardiovascular disease. *Diagnostics*.

